# IL-32 Promotes the Radiosensitivity of Esophageal Squamous Cell Carcinoma Cell through STAT3 Pathway

**DOI:** 10.1155/2021/6653747

**Published:** 2021-02-17

**Authors:** Zhiyu Ma, Zhen Dong, Dingyue Yu, Mingchen Mu, Wanwen Feng, Jiayi Guo, Beibei Cheng, Jiayou Guo, Jianxin Ma

**Affiliations:** ^1^First Department of Radiotherapy, Wanbei Coal-Electricity Group General Hospital, Suzhou, 234000 Anhui, China; ^2^Department of Radiotherapy, BenQ Medical Center Affiliated to Nanjing Medical University, Nanjing, 210000 Jiangsu, China; ^3^Department of Radiotherapy, Bengbu Second People's Hospital Affiliated to Bengbu Medical Collage, Bengbu, 233000 Anhui, China; ^4^Department of Radiotherapy, Lianyungang Municipal Oriental Hospital Affiliated to Bengbu Medical Collage, Lianyungang, 222042 Jiangsu, China; ^5^Translational Medicine Center, Lianyungang Municipal Oriental Hospital Affiliated to Bengbu Medical Collage, Lianyungang, 222042 Jiangsu, China

## Abstract

**Objective:**

This study is set out to determine the relationship between IL-32 and radiosensitivity of esophageal squamous cell carcinoma (ESCC).

**Methods:**

Western blot was adopted for measuring IL-32 expression in Eca-109 and TE-10 cells. Eca-109 and TE-10 cells with interference or overexpression of IL-32 were treated with the presence or absence of X-ray irradiation. Then, the use of CCK8 assay was to detect proliferation ability, and effects of IL-32 expression on radiosensitivity of ESCC were tested by colony formation assay. The cell apoptosis was detected using flow cytometry. STAT3 and p-STAT expression, and apoptotic protein Bax were detected by western blot.

**Results:**

Colony formation assay and CCK8 assay showed that compared with the NC group without treatment, the growth of the ESCC cells, that is Eca-109 and TE-10, was significantly inhibited in the OE+IR group with highly expressed IL-32 and irradiation. In flow cytometry analysis, in Eca-109 and TE-10 cells, highly expressed IL-32 combined with irradiation significantly increased apoptosis compared with the control group. Highly expressed IL-32 has a synergistic effect with irradiation, inhibiting STAT3 and p-STAT3 expression and increasing apoptotic protein Bax expression.

**Conclusion:**

IL-32 can improve the radiosensitivity of ESCC cells by inhibiting the STAT3 pathway. Therefore, IL-32 can be used as a new therapeutic target to provide a new attempt for radiotherapy of ESCC.

## 1. Introduction

About 53% of the new cases of esophageal cancer are esophageal squamous cell carcinoma (ESCC) in the world [1]. At present, comprehensive treatment for esophageal cancer employed radiotherapy as one of the key methods, which mainly includes preoperative radiotherapy, simultaneous radiotherapy and chemotherapy, and postoperative radiotherapy, but the 5-year survival rate (15%-25%) remains unsatisfactory [2]. At present, intensity-modulated radiation therapy (IMRT) is the mainstream radiotherapy for esophageal cancer in the world. This method has been widely studied and applied because of its controllable irradiation range, accurate radiation dose, low dose endangering organs, and low radiation toxicity. Compared with traditional irradiation methods, IMRT has no significant breakthrough in scientific theory but uses radiation to kill cancer cells. The 5-year survival rate has not been significantly improved due to the fact that the tumor cells of esophageal cancer will produce radiotherapy tolerance after multiple radiation exposure [3].

Therefore, it is a critical challenge and of great significance to find an efficient and accurate treatment for esophageal cancer with a breakthrough in scientific theory. Radiotherapy applied in clinical practice mainly aims to improve the radiosensitivity of tumor cells. Cell science has developed by leaps and bounds in recent years, especially at the tumor cell level, revealing the principles of increased radiation tolerance of tumor cells and apoptosis, cell cycle redistribution, high expression of cell genes, and abnormal related signal transduction pathways [4, 5]. The conclusion existed in the study of Zhang et al. regarding miR-519 through PI3K/AKT/mTOR pathway to enhance the radiosensitivity of ESCC cells [6]. As shown in the literature of Yu et al., inhibiting gene expression could also upregulate the radiosensitivity of ESCC cells also [7]. Accordingly, it is of importance to explain the radioresistance mechanism of ESCC, thus improving the sensitivity of radioresistant ESCC cells.

Interleukin 32 (IL-32) is a kind of natural killer cell transcript 4 (NK4) gene product first discovered by Kim et al. [8]. IL-32 can be expressed in a variety of organs or tissues, such as the spleen, thymus, and lung [9]. Heinhuis et al. found that the spatial structure of IL-32 is a typical *α*-helix similar to the adhesion targeting region (FAT) of adhesion kinase (FAK-1). This is the main mechanism of IL-32 in regulating FAT activity and exerting different important biological activities [10]. Previously published studies have confirmed that in TNFR-mediated cells and human melanoma cell line HTB-72 of human IL-32*α* transgenic mouse model, overexpressed IL-32*α* leads to the inhibited cell growth and increased apoptosis [11, 12]. In Jurkat cells and human T cells, overexpressed IL-32 *γ* leads to cell cycle arrest as well as cell death [13]. According to Oh et al.'s research, in human IL-32*γ* overexpression transgenic mice, the continuous activation of STAT3 and NF-*κ*B could be suppressed by IL-32*γ*, thus inhibited the growth of melanoma as well as colon cancer tumors occurring in vitro and in vivo [14]. However, how to further understand the effect of IL-32 gene expression on the radiosensitivity of ESCC is still a great challenge.

The signal transducer and activator of transcription (STAT) family includes STAT3 as one of the most critical members. At present, some studies have shown that STAT3, as a tumor radiosensitivity-related gene, has a clear radioresistant effect. As reported by Aggarwal et al. [15], overexpressed STAT3 could increase the tolerance of head and neck squamous cell carcinoma (SCCHN) cells and nonsmall cell lung cancer (NSCLC) cells to radiation. And the formation of breast cancer radioresistance might also have the participation of STAT3 [16]. In addition, in esophageal cancer, studies have found that after the inhibition of STAT3 activity, radiosensitivity of esophageal cancer cells could be significantly increased [17, 18]. Meanwhile, there is also evidence that IL-32*β* activates the VEGF-STAT3 signal pathway, thereby promoting breast cancer cell migration [19], while inhibits NF-*κ*B and STAT3 signaling pathways to suppress tumor growth [20]. However, the relationship between IL-32 and STAT3 and ECSS radiation resistance needs to be further explored.

The objective of our study is to explain the radioresistant effect of IL-32 and the possible mechanism in ESCC cells in vitro. The present study revealed that upregulated IL-32 can promote the effects of X-ray irradiation (IR) on inhibiting proliferation and increasing apoptosis of ESCC. Furthermore, highly expressed IL-32 suppresses the STAT3 signal pathway, resulting in an increase of the radiosensitivity of ESCC cells. Our experiment helps to find effective targets for ESCC radiosensitization.

## 2. Materials and Methods

### 2.1. Cell Culture and Cell Transfection

Human ESCC lines Eca-109 and TE-10 (Chinese Academy of Sciences in Shanghai, Shanghai, China) were highly differentiated squamous cell carcinoma lines. The cells were cultured in DMEM (Beyotime, Shanghai, China) containing 100 mg/ml streptomycin/penicillin, 10% fetal bovine serum (FBS), and 100 U/ml penicillin in an incubator with 5% CO_2_ at 37°C. IL-32 interference and overexpression lentivirus (Genechem Company, Shanghai, China) were purchased for transfection. After stable transfection, the cells were subcultured and prepared for follow-up experiments.

### 2.2. Irradiation

The cell lines were grouped into the NC group without treatment, the KD group with lowly expressed IL-32, and the OE group with highly expressed IL-32. Subsequently, the cells of each group in the exponential growth phase were treated with IR at doses of 2 Gy, 4 Gy, 6 Gy, and 8 Gy (450 cGy/min).

### 2.3. CCK8 Assay

The cells in the exponential growth phase were made into a 3 × 10^5^/ml cell suspension. A total of 100 *μ*l cell suspension and 100 *μ*l fresh medium were added to the 96-well plate. After 24 hours, 8 Gy X-ray was used to treat the cells of each group for 24, 48, and 72 hours, respectively, and then, CCK8 reagent was added. The absorbance value of each group of cells was detected using a microplate reader (450 nm).

### 2.4. Colony Formation Assay

Six cell lines Eca-109 (NC), TE-10 (NC), Eca-109 (KD), TE-10 (KD), Eca-109 (OE), and TE-10 (OE) were seeded into six-well plates at 1000 cells per well. At 24 hours after culture, cells were treated with IR at 0 Gy, 2 Gy, 4 Gy, 6 Gy, and 8 Gy. At 6 hours after IR, following the change of fresh culture medium, the culture was continued for 12 days. On completion of 15 min fixation using 4% paraformaldehyde, 0.1% crystal violet was adopted for 20 min staining. Under a light microscope, 50 or more colonies were counted. Survival fraction (SF) = number of colonies formed ÷ number of coated cells. The GraphPad Prism 8.0 software was applied to fit cell survival curves and radiation biological parameters, including D0 (final slope), Dq (quasi-threshold dose), SF2 (2 Gy of SF), and SER (sensitization enhancement ratio).

### 2.5. Flow Cytometry

Prior to exposure to therapy dose of 8 Gy, the cells were cultured overnight at 37°C in 6-well plates (1 × 10^5^ cells/well). At 24 hours after culture, Annexin V-FITC (BD Bioscience, Oxford, UK) and PI were employed for staining. Finally, flow cytometry was adopted to detect cell apoptosis based on their light scatter property.

### 2.6. Western Blot

After IR, the RIPA lysis buffer was used to lyse the cells. After the protein concentration was confirmed by the BCA protein detection kit (Beyotime, Shanghai, China), the proteins of the same concentration were separated using 10% SDS-PAGE and then transferred to PVDF membrane (Millipore, USA). Following the blocking step using 5% milk, antibodies were added to the membranes overnight at 4°C, including IL-32 antibody from Proteintech, USA, and STAT3 antibody, p-STAT3 antibody, Bax antibody, and GAPDH antibody from Cell Signaling Technology, USA. Subsequently, the membranes were incubated with the secondary antibodies (Cell Signaling Technology, USA) at room temperature for 2 hours. Immunoblotting protein was detected by enhanced chemiluminescence.

### 2.7. Network Gene Analysis

Based on publicly available biological data sets, the association between the IL-32 genes and other genes was analyzed using GEPIA (http://gepia.cancer-pku.cn/).

### 2.8. Statistical Analysis

The statistical analyses were performed using the SPSS software (version 22.0). The data were expressed in the form of mean ± standard deviation (SD). Student's*t*-test was adopted for comparison between two groups. Each experiment was repeated at least three times. Differences were considered statistically significant if *P* < 0.05.

## 3. Result

### 3.1. Expression Efficiency of IL-32

The expression efficiency was tested by western blot after transfection of IL-32 overexpression or interference lentivirus. As can be seen from Figure 1, after transfection with IL-32 interference lentivirus, the protein expression of IL-32 was downregulated, while upregulated after transfection with IL-32 overexpression lentivirus. The results confirmed that the IL-32 expression in ESCC was interfered successfully.

### 3.2. High Expression of IL-32 Inhibits ESCC Cell Proliferation after Irradiation

Drawing upon the aim of detection of the effect of IL-32 on the radiosensitivity of ESCC cells at the cellular level, the CCK8 assay was adopted for testing proliferation. Each group received 8 Gy IR, and the OD values were measured at 24, 48, and 72 h, respectively. The results showed that both IR and upregulated IL-32 could inhibit proliferation. In comparison with the IR group, this inhibitory effect was promoted in the OE+IR group (*P* > 0.05) (Figures 2(a) and 2(b)).

In addition, the colony formation assay revealed that in the OE group, the SF values of Eca-109 and TE-10 (Figure 3) of different doses of X-rays were lower than the NC group. Compared with the NC group, the D0 (1.85 vs. 2.84 and 2.15 vs. 2.34) and Dq (0.46 vs. 0.71 and 0.3 vs. 1.19) in the OE groups were significantly lower. However, the values of D0 and Dq in the KD group did not change significantly (Table 1 and Table 2). Furthermore, as shown in Figure 4, in comparison with the NC group, the clone formation ability in the OE group was decreased after 2 Gy IR, while it was increased in the KD group. It can be indicated that highly expressed IL-32 led to a significant increase in radiosensitivity of ESCC cells.

### 3.3. High Expression of IL-32 Promotes ESCC Cell Apoptosis after Irradiation

Apoptosis is one of the main mechanisms of tumor cell death. The Eca-109 and TE-10 cells were detected for apoptosis in the presence or absence of 8 Gy IR (Figure 5). Both IR and upregulated IL-32 could promote apoptosis. In comparison with the IR group, cell apoptosis in the OE+IR group was significantly increased (Figure 5). It can be suggested that upregulated IL-32 promoted apoptosis and enhanced the ESCC radiosensitivity.

### 3.4. High Expression of IL-32 Promotes the Inhibitory Effect of Irradiation on STAT3 Activation in ESCC Cells

Further experiments on the molecular mechanism by which IL-32 affects the radiosensitivity of ESCC cells were carried out. First of all, the related genes were analyzed on the Internet, and the data obtained were set out a positive correlation of the IL-32 expression and apoptotic proteins Bax and Bak1 (Figure 6). Next, the protein expression levels of Bax, STAT3, and p-STAT3 were detected. Western blot revealed that when exposed to IR (8 Gy), compared with the NC and KD group, STAT3 and p-STAT3 protein expression in the OE group was significantly downregulated, and Bax was significantly upregulated (Figures 7(a) and 7(b)).

## 4. Discussion

Esophageal cancer has no obvious clinical symptoms in the early stage. Patients occurring typical symptoms such as progressive dysphagia or choking basically belong to the middle and advanced stage and may lose the opportunity of operation [21, 22]. In addition, the operation of cervical esophageal cancer is quite difficult, and preoperative radiotherapy is also widely used, so radiotherapy is one of the key means for esophageal cancer treatment [23]. Tumor cells activate cytotoxic reactions after radiation, resulting in DNA damage. But like other cells, tumor cells will activate complex detection and repair mechanisms to avoid radiation-induced cell death, that is, initiating cell cycle arrest and attempting to repair apoptosis in the event of major damage [24].

Downregulation of IL-32 protein expression has been reported to cause a decrease in human KG1a leukemia cells and an imbalance of inflammatory cytokines [25]. Other studies have shown that miR-205 increases IL-32 expression and is involved in prostate cancer cell apoptosis, increased migration, and decreased invasion [26]. Some reports also support that IL-32 inhibits the growth of colorectal cancer cells and tumor, indicating that IL-32*γ* can upregulate the p32-MAPK signal to enhance TNF-*α*-mediated cell apoptosis [27]. These studies indicate that IL-32 may have antitumor effects. In our current research, we found that in Eca-109 and TE-10 cells, both IR and high expression IL-32 could lead to inhibition of proliferation and clone formation, and promotion of apoptosis. Meanwhile, highly expressed IL-32 could further promote the effects of IR. In addition, the gene analysis data based on the network presented that the IL-32 expression had a positive correlation with Bax and Bak1. Western blot also confirmed that overexpression of IL-32 and IR could promote the expression of Bax protein in Eca-109 and TE-10 cells, and ESCC cells with high IL-32 expression have higher Bax protein expression after IR exposure. These results confirm that highly expressed IL-32 can increase the radiosensitivity of ESCC cells.

Many published literature has proved that STAT3 has a carcinogenic effect, and STAT3 is activated in many solid tumors and hematological tumors [28–31]. Generally speaking, continuously activated STAT3 produces a signal input to the tumor, thus protecting tumor cells from apoptosis [32]. STAT3 has been studied as the intersection of many carcinogenic signal pathways due to its effects in tumor cells and tumor microenvironment. In lung cancer cells, including NSCLC, an association was found between STAT3 activation and phosphorylation and increased cell proliferation, angiogenesis, and metastasis [33]. In human hepatocellular carcinoma (HCC) samples, phosphorylated STAT3 was found [34]. Colorectal cancer has shown an obvious active state of STAT3 signal pathway [35] and with strongly expressed STAT3 in tumor cells and infiltrating lymphocytes [36]. Patients with gastric cancer have poor STAT3 protein activation and survival prognosis [37]. In this study, STAT3 and p-STAT3 protein expression was downregulated by upregulated IL-32 or 8Gy IR. In addition, Eca-109/TE-10 cells with high IL-32 expression had lower STAT3 and p-STAT3 protein expression after IR. It is suggested that STAT3 expression and phosphorylation are inhibited by IR, and this inhibitory effect is further promoted by highly expressed IL-32.

In summary, upregulation of IL-32 can improve the radiosensitivity of ESCC by inhibiting the STAT3 signal pathway. IL-32 can be used as a new therapeutic target, providing a new attempt for radiotherapy of ESCC. Since there are many subtypes of IL-32, studies are still required to further clarify the specific molecular mechanism of the radiation effect of various subtypes of IL-32 on ESCC cells in the future.

## Figures and Tables

**Figure 1:** Western blot was used to detect the expression efficiency of IL-32. KD: low expression of IL-32; OE: overexpression of IL-32.

**Figure 2:** The IL-32 overexpression inhibits ESCC proliferation and synergistically improves radiosensitivity. The Eca-109 (a) and TE-10 cells (b) in each group were irradiated with 8 Gy X-ray, and the OD values were measured by CCK8 assay at 24, 48, and 72 hours, respectively. ^∗∗^*P* < 0.01. KD: low expression of IL-32; OE: overexpression of IL-32; IR: X-ray irradiation.

**Figure 3:** Colony formation was used to detect survival curves. KD: low expression of IL-32; OE: overexpression of IL-32.

**Figure 4:** Effect of IL-32 expression on the clonogenic ability after 8 Gy X-ray irradiation. KD: low expression of IL-32 expression; OE: overexpression of IL-32.

**Figure 5:** Effect of IL-32 overexpression on Eca-109 and TE-10 cell apoptosis after 8 Gy X-ray irradiation. The data obtained from three independent flow cytometry analyses are expressed in the form of mean ± standard deviation (SD). ^∗∗^*P* < 0.01. OE: overexpression of IL-32; IR: X-ray irradiation.

**Figure 6:** Network-based gene analysis showed a correlation between IL-32 expression and apoptotic proteins Bax and Bak1.

**Figure 7:** Upregulation of IL-32 inhibits STAT3 activation. In the KD and OE groups, Bax, p-STAT3, and STA T3 protein expression was measured by western blot in Eca-109 (a) and TE-10 (b) cells in the presence or absence of 8 Gy X-ray irradiation. KD: low expression of IL-32; OE: overexpression of IL-32; IR: X-ray irradiation.

**Table 1:** Radiosensitization of IL-32 in Eca-109 cells.

	D0 (Gy)	Dq (Gy)	SF2	SER
KD	2.81	1.04	0.59	1.01
NC	2.84	0.71	0.56	
OE	1.85	0.46	0.41	1.54

Data are presented as the slope of the curve fitted. The radiation biologic parameters were calculated by GraphPad Prism 8.0 that was fitted into the single-hit multitarget formula:SF = 1 − (1 − exp(−*k* × *x*))^*N*^;*k* = 1/D0;ln*N* = Dq/D0;SER = D0 (control group)/D0 (experimental group). D0: final slope; Dq: quasi-threshold dose; SF2: 2 Gy of survival fraction (SF); SER: sensitization enhancement ratio; KD: low IL-32 expression; OE: overexpression IL-32.

**Table 2:** Radiosensitization of IL-32 in TE-10 cells.

	D0 (Gy)	Dq (Gy)	SF2	SER
KD	2.49	1.69	0.63	0.94
NC	2.34	1.19	0.57	
OE	2.15	0.3	0.40	1.09

Data are presented as the slope of the curve fitted. The radiation biologic parameters were calculated by GraphPad Prism 8.0 that was fitted into the single-hit multitarget formula: SF = 1 − (1 − exp(−*k* × *x*))^*N*^; *k* = 1/D0; ln*N* = Dq/D0; SER = D0 (control group)/D0 (experimental group). D0: final slope; Dq: quasi-threshold dose; SF2: 2 Gy of survival fraction (SF); SER: sensitization enhancement ratio; KD: low IL-32 expression; OE: overexpression IL-32.

## Data Availability

Some or all data, models, or code generated or used during the study are available from the corresponding author by request.

## References

[1] Arnold M., Soerjomataram I., Ferlay J., Forman D. (2015). Global incidence of oesophageal cancer by histological subtype in 2012. *Gut*.

[2] Enzinger P. C., Mayer R. J. (2003). Esophageal cancer. *New England Journal of Medicine*.

[3] Kurtom S., Kaplan B. J. (2020). Esophagus and gastrointestinal junction tumors. *The Surgical clinics of North America*.

[4] Letai A. (2017). Apoptosis and cancer. annual review of cancer biology.

[5] Krammer P. H., Weyd H. (2017). Life, death and tolerance. *Biochemical and Biophysical Research Communications*.

[6] Zhang Y., Chen W., Wang H., Pan T., Zhang Y., Li C. (2019). Upregulation of miR-519 enhances radiosensitivity of esophageal squamous cell carcinoma trough targeting PI3K/AKT/mTOR signaling pathway. *Cancer Chemotherapy and Pharmacology*.

[7] Yu D., Ma Y., Feng C. (2020). PBX1 Increases the radiosensitivity of oesophageal squamous cancer by targeting of STAT3. *Pathology & Oncology Research: Official Journal of the Arányi Lajos Foundation*.

[8] Kim S. H., Han S. Y., Azam T., Yoon D. Y., Dinarello C. A. (2005). Interleukin-32: a cytokine and inducer of TNFalpha. *Immunity*.

[9] Joosten L. A. B., Heinhuis B., Netea M. G., Dinarello C. A. (2013). Novel insights into the biology of interleukin-32. *Cellular and Molecular Life Sciences*.

[10] Heinhuis B., Koenders M. I., van Riel P. L. (2011). Tumour necrosis factor alpha-driven IL-32 expression in rheumatoid arthritis synovial tissue amplifies an inflammatory cascade. *Annals of the Rheumatic Diseases*.

[11] Nicholl M. B., Chen X., Qin C. (2016). IL-32*α* has differential effects on proliferation and apoptosis of human melanoma cell lines. *Journal of Surgical Oncology*.

[12] Yun H.-M., Park K.-R., Kim E.-C., Han S. B., Yoon D. Y., Hong J. T. (2015). IL-32*α* suppresses colorectal cancer development via TNFR1-mediated death signaling. *Oncotarget*.

[13] Goda C., Kanaji T., Kanaji S. (2006). Involvement of IL-32 in activation-induced cell death in T cells. *International Immunology*.

[14] Oh J. H., Cho M.-C., Kim J.-H. (2011). IL-32*γ* inhibits cancer cell growth through inactivation of NF-*κ*B and STAT3 signals. *Oncogene*.

[15] Aggarwal B. B., Sethi G., Ahn K. S. (2007). Targeting Signal-transducer-and-activator-of-transcription-3 for prevention and therapy of cancer: modern target but ancient solution. *Annals of the New York Academy of Sciences*.

[16] Kim J.-S., Kim H.-A., Seong M.-K. (2016). STAT3-survivin signaling mediates a poor response to radiotherapy in HER2-positive breast cancers. *Oncotarget*.

[17] Zhang C., Yang X., Zhang Q. (2014). STAT3 inhibitor NSC74859 radiosensitizes esophageal cancer via the downregulation of HIF-1*α*. *Tumor Biology*.

[18] Zhang Q., Zhang C., He J. (2015). STAT3 inhibitor stattic enhances radiosensitivity in esophageal squamous cell carcinoma. *Tumour biology : the journal of the International Society for Oncodevelopmental Biology and Medicine*.

[19] Park J. S., Choi S. Y., Lee J.-H. (2013). Interleukin-32*β* stimulates migration of MDA-MB-231 and MCF-7cells via the VEGF-STAT3 signaling pathway. *Cellular Oncology*.

[20] Yun H.-M., Oh J. H., Shim J.-H. (2013). Antitumor activity of IL-32*β* through the activation of lymphocytes, and the inactivation of NF-*κ*B and STAT3 signals. *Cell Death & Disease*.

[21] Tirumani H., Rosenthal M. H., Tirumani S. H., Shinagare A. B., Krajewski K. M., Ramaiya N. H. (2015). Esophageal carcinoma: current concepts in the role of imaging in staging and management. *Canadian Association of Radiologists Journal*.

[22] Ohashi S., Miyamoto S.’i., Kikuchi O., Goto T., Amanuma Y., Muto M. (2015). Recent advances from basic and clinical studies of esophageal squamous cell carcinoma. *Gastroenterology*.

[23] Shridhar R., Almhanna K., Meredith K. L. (2013). Radiation therapy and esophageal cancer. *Cancer Control : journal of the Moffitt Cancer Center*.

[24] Arnoult N., Correia A., Ma J. (2017). Regulation of DNA repair pathway choice in S and G2 phases by the NHEJ inhibitor CYREN. *Nature*.

[25] Marcondes A. M., Mhyre A. J., Stirewalt D. L., Kim S.-H., Dinarello C. A., Deeg H. J. (2008). Dysregulation of IL-32 in myelodysplastic syndrome and chronic myelomonocytic leukemia modulates apoptosis and impairs NK function. *Proceedings of the National Academy of Sciences of the United States of America*.

[26] Majid S., Dar A. A., Saini S. (2010). MicroRNA-205–directed transcriptional activation of tumor suppressor genes in prostate cancer. *Cancer*.

[27] Park E.-S., Yoo J.-M., Yoo H.-S., Yoon D.-Y., Yun Y.-P., Hong J. T. (2014). IL-32*γ* enhances TNF-*α*-induced cell death in colon cancer. *Molecular Carcinogenesis*.

[28] Zhang H. F., Lai R. (2014). STAT3 in cancer—friend or foe?. *Cancers*.

[29] Eirini B., Jacqueline B. (2013). Targeting the tumor microenvironment: JAK-STAT3 signaling. *JAK-STAT*.

[30] Avalle L., Pensa S., Regis G., Novelli F., Poli V. (2012). STAT1 and STAT3 in tumorigenesis: a matter of balance. *JAK-STAT*.

[31] Sellier H., Rébillard A., Guette C., Barré B., Coqueret O. (2013). How should we define STAT3 as an oncogene and as a potential target for therapy?. *JAK-STAT*.

[32] Bowman T., Garcia R., Turkson J., Jove R. (2000). STATs in oncogenesis. *Oncogene*.

[33] Harada D., Takigawa N., Kiura K. (2014). The role of STAT3 in non-small cell lung cancer. *Cancers*.

[34] He G., Karin M. (2011). NF-*κ*B and STAT3 - key players in liver inflammation and cancer. *Cell Research*.

[35] Park J. H., van Wyk H., McMillan D. C. (2017). Signal transduction and activator of transcription-3 (STAT3) in patients with colorectal cancer: associations with the phenotypic features of the tumor and host. *Clinical Cancer Research*.

[36] Lin L., Liu A., Peng Z. (2011). STAT3 is necessary for proliferation and survival in colon cancer–initiating cells. *Cancer Research*.

[37] Chai E. Z. P., Shanmugam M. K., Arfuso F. (2016). Targeting transcription factor STAT3 for cancer prevention and therapy. *Pharmacology & Therapeutics*.

